The article "The Expression Profile of miRNA in Glioma and the Role of miR-339-5p in Glioma" was retracted in 2024. Reasons: signs of a paper mill; suspected computer-generated content; unreliable results or conclusions; concerns about the data.

# The Expression Profile of miRNA in Glioma and the Role of miR-339-5p in Glioma

**DOI:** 10.1155/2022/4085039

**Published:** 2022-06-22

**Authors:** Jie Lin, Shouyi Wang, Huanan Shen, Buyi Zheng

**Affiliations:** ^1^Department of Neurosurgery, Wenzhou People's Hospital, Wenzhou, Zhejiang Province, China 325000; ^2^Department of Vascular & Interventional Radiology, Wenzhou People's Hospital, Wenzhou, Zhejiang Province, China 325000; ^3^Department of Neonatology, Wenzhou People's Hospital, Wenzhou, Zhejiang Province, China 325000

## Abstract

**Objective:**

To reveal the expression profile of miRNA in glioma and the effects of microRNA-339-5p (miR-339-5p) on glioma.

**Methods:**

The glioma and normal tissues were randomly selected for miRNA gene chip detection and qRT-PCR verification. The U87 cells were separated into miR-NC, miR-339-5p mimic, and miR-339-5p suppressor group. Clonogenesis test, flow cell technique, Transwell, and cell scratch assay were utilized to verify the roles of miR-339-5p in cell proliferation, cell apoptosis, cell invasion, and cell migration. The epithelial-meso-transformation-associated proteins was verified by Western blot.

**Results:**

A total of 49 miRNAs (16 upregulated and 33 downregulated) were differentially expressed in glioma tissues, and miR-339-5p was the most downregulated. The clone number, invasion number, and healing rate of cells in miR-339-5p mimic group were decreased compared with miR-NC group (*P* < 0.05); the clone quantity, invasion number, and healing rate of cells in miR-339-5p inhibitor group were increased compared with miR-NC group (*P* < 0.05). The apoptosis rate of human glioma U87 cells in miR-339-5P mimic group was compared with miR-NC group (*P* < 0.05); the apoptosis rate of human glioma U87 cells in miR-339-5p suppressor group decreased compared with miR-NC group (*P* < 0.05). Compared with miR-NC group, the protein expression of Twist, Snsnail, N-cadherin, and Vimentin in miR-339-5p mimic group was considerably decreased, whereas E-cadherin was elevated (*P* < 0.05). Compared with miR-NC group, the protein expression of Twist, Snsnail, N-cadherin, and Vimentin in miR-339-5p suppressor group was considerably increased, whereas E-cadherin was considerably decreased (*P* < 0.05).

**Conclusion:**

Forty-nine glioma-related miRNAs were screened out, and miRNA expression was significantly different between glioma and normal tissues. The downregulated miR-339-5p in glioma can regulate the proliferative, apoptotic, invasive, and migratory abilities of glioma U87 cells and might suppress the occurrence and development of glioma.

## 1. Introduction

Tumors originating from neuroepithelium are collectively referred to as glioma, which is caused by the canceration of glial cells in the cerebrum and spinal cord and is featured by obvious invasiveness, high morbidity, and high death rate [1]. The pathogenic factors of this disease are relatively complex. Under the interaction of congenital genetic factors and environmental carcinogenic factors, the level of genetic and epigenetic material of cells has undergone cancer mutation [2]. These mutations drive cells to continuously enter the cell cycle, avoid immune suppression, apoptosis, and mitosis, and contact suppression of cell growth, etc., and abnormal energy metabolism, hypoxia, and necrosis corresponding to continuous cell growth also induce changes in tumor angiogenesis [3]. Low-grade gliomas develop slowly and have a good clinical prognosis, while high-grade gliomas develop rapidly and have a poor clinical prognosis [4]. Due to the rapid growth rate and high infiltration of glioma, the blood-brain barrier restriction cannot allow anticancer drugs to enter the central nervous system [5], and the effect of surgery combined with radiotherapy and chemotherapy is not satisfactory. Hence, it is imperative to identify the etiopathogenesis of glioma, search for biomarkers for diagnosis and treatment, and screen therapeutic targets for prolonging the survival of patients. miRNAs are highly conserved and are pivotal for gene expression, translation, and posttranscriptional regulation of biological processes [6]. MicroRNAs (miRNAs) have drawn much attention because of their diagnostic value in diverse cancers, including glioma. The exchange of miRNAs through gap junctions has been reported between glioma cells and from mesenchymal stem cells to glioma cells. It extensively participates in physiopathological process like tissue differentiation, neural development, synaptic formation, and cell apoptosis [7]. Current studies have shown that miRNA is tightly associated with the onset and developmental process of glioma. However, the role of miR-339-5p in glioma remains unknown. In the present study, we first detected the expression of miR-339-5p in glioma. The regulatory effect of miR-339-5p on glioma was further explored. In this paper, our team identified the expression profile of miRNA in the brain tissue of glioma patients and investigated the roles of miR-339-5p in the pathogenesis of glioma. The specific report is as follows.

## 2. Materials and Methods

### 2.1. Total RNA Extraction

Overall RNA was abstracted from tissues via TRIzol (Qiagen, Valencia, CA). Glioma tissues and normal tissues were ground into powder in liquid nitrogen, mixed with TRIzol, and centrifuged at 4°C at 12000 × *g* for 5 min, then the supernate was moved to a novel EP tube of chloroform and isoamyl alcohol, and the centrifugation was continued. After centrifugation, the upper RNA was taken and washed with ethanol, the ethanol was removed, and the RNA was dissolved in DEPC water. The total RNA was identified and quantified by NanoDrop and Agilent 2100 bioanalyzer.

### 2.2. miRNA Gene Chip Detection and Analysis

A total of 50 patients with glioma (age range, 39-80 years; mean age, 59 years) were diagnosed between January 2021 and June 2022 at Wenzhou People's Hospital. Ten glioma tissues and 10 normal tissues were randomly selected for miRNA chip detection. After total RNA extraction, miRNA was labeled; total RNA, CIP buffer, and CIP enzyme were mixed with a centrifuge tube without RNA enzyme; PCR cycle was conducted; and CIP was added. The reaction was performed after 5 step: labeling buffer, fluorescent label (Hy3 TM), DMSO, labeling enzyme, and mixing; PCR cycle was conducted once; and miRNA chip hybridization was performed 24 h later. Exiqon miRCURY™ LNA Array (V.18.0) chip was used to detect miRNA expression in the tissues of the above two groups.

### 2.3. qRT-PCR Was Used to Verify miRNAs

After total RNA extraction, total RNA absorbance was determined, and cDNA was retrotranscribed as per the specification of the miRcute miRNA fluorescent quantitation identification tool. PCR reaction system was 25 *μ*L, TB Green Premix Ex Taq II 12.5 *μ*L (Bio-Rad), PCR Forward Primer 1 *μ*L (Bio-Rad), PCR Reverse Primer 1 *μ*L (Bio-Rad), cDNA 2 *μ*L (Bio-Rad), and RNase Free dH2O 8.5 *μ*L; reactive conditions are as follows: predenaturation under 95°C for 0.5 min, denaturized under 95°C for 5 s, and annealing and extension under 60°C for 0.5 min, an overall 40. The CT value of 2-*ΔΔ*CT was calculated as the comparative expression value of the gene according to the CT result of the targeted gene in each specimen. The following primer pairs were used for the qPCR: miR-339-5p forward: 5′-GCCGAGTCCCTGTCCTCCAGG-3′ and reverse: 5′-CTCAACTGGTGTCGTGGA-3′ and U6 forward: 5′-GCTTCGGCAGCACATATACTAAAAT-3′ and reverse: 5′-CGCTTCACGAATTTGCGTGTCAT-3′.

### 2.4. Cell Culture and Grouping

Human glioma U87 cells were cultivated with RPMI 1640 intermediary involving 10% FBS and 1 × 105 U/L penicillin/streptomycin dual antibody solution in a constant temperature incubator. Follow-up experiments were carried out when the cells were in log-growth phase. U87 cells were separated into miR-NC group, miR-339-5p mimic group, and miR-339-5p suppressor group. The cells in every group were inoculated into 6-well dishes, and Lipofectamine 3000 was transfected, and strict operations were completed as per the supplier's specification. miR-nc was introduced into U87 cells via transfection as miR-NC group. miR-339-5p mimic was introduced into U87 cells via transfection, and miR-339-5p suppressor was introduced into U87 cells via transfection and miR-339-5p suppressor was introduced into U87 cells via transfection. Transfection efficiency values were obtained through measurements after cell-lysis activity assay and were compared to efficiencies obtained in parallel with a commercially available liposome-preparation (Lipofectamine).

### 2.5. The Proliferative Ability of U87 Cells Was Detected by Clonal Formation Assay

U87 cells in every group at log-growth phase were subjected to digestion via trypsin to produce cellular suspension, and the cellular density was adjusted to 2.0 × 10^3^ cells/cell. The culture medium was discarded, the culture medium was cleaned with PBS, methanol was added and fixed for 15 min, PBS was cleaned, crystal violet staining was performed for 20 min, PBS was rinsed, and photography was counted.

### 2.6. Apoptosis of U87 Cells Was Identified by Flow Cell Technique

Posterior to the 48 h transfectional process, the cells were cleaned in PBS and prepared into suspension. Annexin V-FITC 5 *μ*L and 5 *μ*L PI (Thermo Fisher Scientific) were supplemented into the suspension under dark conditions. The cells were cultivated for 15 min and analyzed by flow cell technique to identify apoptosis rate of U87 cells in every group.

### 2.7. U87 Cell Invasion Was Detected by Transwell

An appropriate amount of diluted Matrigel was supplemented into Transwell chamber (Beckman Coulter, Fullerton, CA) and cultivated with 5% CO_2_ and 37°C culture phase until the matrix gelated. The cells were prepared into suspension and seeded into a 24-well dish with 5 × 10^4^ cells per well, incubated at room temperature for 24 h, subjected to fixation in methyl alcohol for 0.5 h, dyed in 0.1% gentian violet for 20 min, washed with water, and removed the cells that did not penetrate the membrane. The cells were observed under microscope in 5 fields and photographed for counting.

### 2.8. Cell Scratch Test U87 Cell Migration

U87 cells in each group were transfected with liposome (Millipore) for 48 h, and the cellular content was modified to 1 × 10^6^ cells/dish. The cells were seeded in a 35 mm Petri dish, added to the medium, and cultivated in a 5% CO_2_ incubating device under 37°C. After discarding the intermediary, PBS was used for cleaning, 200 *μ*L spear tip was used to uniformly make linear scratches in the Petri dish, and the scratches in each group were roughly the same in thickness. PBS was used to wash the scratch healing area, then intermediary without serum was added, and pictures were captured via a microscopic device, which was marked as 0 h. Culture and incubation were continued, and images were taken under the microscope at 48 h.

### 2.9. The Expression of Epithelial-Mesenchymal (E-M) Transformational Proteins Was Identified via Western Blot

All reagents were obtained from Sigma-Aldrich (St. Louis, MO). The transfected U87 cells of each group were used for ice lysis with cell lysate containing PMSF, and protein was collected. Protein levels were identified via BCA approach and SDS-PAGE polyacrylamide gel electrophoresis, closed, incubation Twist (1 : 500), snq-2 (1 : 1000), N-cadherin (1 : 500), Vimentin (1 : 1000), E-cadherin (1 : 500) primary antibody, 4°C shaking bed overnight. HRP labeled second antibody (1 : 10,000) was cultivated for 120 min, the membrane was removed and cleaned with TBST, and ECL luminescent solution was added for exposure, and pictures were taken.

### 2.10. Statistical Treatment

GraphPad Prism 9 was utilized for statistic assay, and data was represented by $\bar{x}\pm s$. *T*-test was utilized for pair-to-group contrast, and ANOVA was utilized for multigroup contrast. *P* < 0.05 had significance on statistics.

## 3. Results

### 3.1. Analysis of Quality and Quantity of RNA Samples

The A260/A280 of the extracted RNA was in the range of 1.8~2.1, with good RNA purity and no obvious degradation, and no protein contamination during the extraction process, which can be used for subsequent experiments.

### 3.2. Microarray Expression Profile of miRNA in Glioma

The microarray hybridization results were analyzed, and the analysis standards were set as follows: multiple of change ≥2 and *P* ≤ 0.05 were considered as differential expression. Compared with normal tissues, 49 miRNAs were differentially expressed in glioma tissues, of which 16 miRNAs were upregulated, 33 miRNAs were significantly downregulated, and the downregulation of miR-339-5p was the most remarkable in the differential expression spectrum. miR-339-5p was chosen as the object of subsequent research. The heat map results of the 49 differentially expressed miRNA are shown in Figure 1 and Table 1.

### 3.3. Validation of miRNAs by qRT-PCR

Based on miRNA chip screening, miR-339-5p with low expression was selected as research objects, and qRT-PCR was utilized to detect 8 miRNAs. The outcomes revealed that the expression of miR-339-5p, miR-185, and miR-539 in glioma was lower than those in healthy samples, and the diversities displayed significance on statistics (*P* < 0.05); qRT-PCR outcomes reveal that the chip results can be trusted, as shown in Figure 2.

### 3.4. Role of miR-339-5p in the Proliferative Ability of Human Glioma U87 Cells

The outcomes revealed that the number of human glioma U87 cells cloned in miR-339-5p mimic group was considerably smaller vs. miR-NC group, and the diversities displayed significance on statistics (*P* < 0.05), the clone quantity of human glioma U87 cells in miR-339-5p suppressor group was considerably greater vs. miR-NC group, and the diversities displayed significance on statistics (*P* < 0.05), as presented by Figure 3.

### 3.5. Role of miR-339-5p in the Programmed Cell Death of Human Glioma U87 Cells

Flow cell technique revealed that the apoptotic rate of HUMAN glioma U87 cells in miR-339-5p mimic group was considerably greater vs. miR-NC group, and the diversity displayed significance on statistics (*P* < 0.05), the apoptotic rate of human glioma U87 cells in miR-339-5p suppressor group was considerably lower vs. miR-NC group, and the diversity displayed significance on statistics (*P* < 0.05), as presented by Figure 4.

### 3.6. Roles of miR-339-5P in Invasion of Human Glioma U87 Cells

Transwell outcomes revealed that the invasion quantity of mankind glioma U87 cells in miR-339-5p mimic group was considerably smaller vs. miR-NC group, and the diversity displayed significance on statistics (*P* < 0.05), the invasion quantity of human glioma U87 cells in miR-339-5p suppressor group was considerably greater vs. miR-NC group, and the diversity displayed significance on statistics (*P* < 0.05), as presented by Figure 5.

### 3.7. Roles of miR-339-5P in Human Glioma U87 Cell Migration

The outcomes of cell scratch assay revealed that the healing rate of human glioma U87 cells in miR-339-5p mimic group was significantly lower vs. miR-NC group, the difference had significance on statistics (*P* < 0.05), the healing rate of human glioma U87 cells in miR-339-5p suppressor group was considerably greater vs. miR-NC group, and the difference had significance on statistics (*P* < 0.05), as presented by Figure 6.

### 3.8. Role of miR-339-5P in E-M Transformation-Associated Proteins in Human Glioma U87 Cells

Western blot revealed that miR-339-5p was considerably higher vs. the miR-nc group, and the protein expression levels of Twist, Snake-2, N-cadherin, and Vimentin were reduced considerably in mimic group, whereas the protein expression level of E-cadherin increased considerably (*P* < 0.05). In contrast to miR-NC group, the protein expression levels of Twist, Snsnail, N-cadherin, and Vimentin in miR-339-5p suppressor group was considerably increased, whereas the protein expression level of E-cadherin was considerably reduced (*P* < 0.05), as presented by Figure 7.

## 4. Discussion

miRNA is an endogenetic noncoding RNA with regulatory function, which is widely involved in various physiological processes of cells, organogenesis, and the development of organisms [8]. Many research has revealed that miRNAs can modulate the onset, progression, and metastases of cancers and become markers and therapeutic targets of related tumors [9], thus providing possibilities for tumor diagnosis and treatment. Related studies have analyzed miRNA expression profiles in cancer and healthy samples at different stages and found that miRNA can distinguish between cancer and healthy samples [10]. miRNA is widely found in gliomas, but the expression levels of each miRNA are different in gliomas [11]. Relevant studies used real-time fluorescent quantification PCR reaction to identify the expression levels of 10 miRNAs in malignant tumors of different degrees and found that the higher the malignant degree of glioma, the lower the expression levels of miR-137 and miR-7, and miR-21, miR-17, miR-9, miR-26a, miR-23a, and miR-20a were subsequently increased [12]. Piwecka et al. demonstrated that miRNA differential expression may be an important molecular biomarker for gliomas and has potential research value in gene expression regulation [13]. Therefore, some miRNAs with abnormal expression in glioma tissues are pivotal for the etiopathogenesis of glioma.

Herein, gene chip technology was used to detect miRNAs, and a total of 49 miRNAs displayed different expression in glioma tissues, 16. The expression levels of 33 miRNAs were considerably upregulated, and the expression of 33 miRNAs was significantly downregulated. qRT-PCR was completed to verify the differentially sequenced miRNAs, and the outcomes revealed that the expression of miR-339-5p, miR-185, and miR-539 in glioma was lower than that in normal samples, and miR-339-5p was regulated downward most obviously. There are few reports about miR-339-5p in gliomas, and recent researchers have found that miR-339-5p is abnormally expressed in many solid tumors. Relevant research has revealed that miR-339-5p is regulated downward in pulmonary carcinoma lineage cells [14], and miR-339-5p is regulated downward in colonic carcinoma tissular specimens and colonic carcinoma lineage cells [15]. In the present paper, the role of miR-339-5p in the proliferative, apoptotic, invasive, and migratory abilities of human glioma U87 cells was demonstrated. The outcomes revealed that the number of clones, invasion, and healing rate of human glioma U87 cells subjected to miR-339-5p mimic transfection were considerably smaller vs. cells subjected to miR-NC and miR-339-5P transfection. The cloning quantity, invasive quantity, and healing rate of human glioma U87 cells in the suppressor group were considerably greater vs. cells in the miR-NC transfection group. The apoptosis rate of human glioma U87 cells subjected to miR-339-5p mimic transfection was evidently smaller in contrast to cells subjected to miR-NC transfection, and the apoptosis rate of human glioma U87 cells subjected to miR-339-5p suppressor transfection was considerably smaller in contrast to cells subjected to miR-NC transfection. Those outcomes reveal that overly expressed miR-339-5p can suppress the proliferative, invasive, and migratory abilities of human glioma U87 cells and facilitate programmed cell death and suppress the expression of miR-339-5p on the contrary. Relevant research has revealed that miR-339-5P suppresses the migratory and invasive abilities of non-small-cell oncocytes and is closely related to cancer lymphatic metastases phase and lymphonodus metastases [16]. Other studies have shown that suppression of miR-339-5p expression elevated the migratory and invasive abilities of OVCAR5 cells, whereas in SKOV3 cells, upregulated miR-339-5P weakened the migratory and invasive abilities [17], like the results of this study.

Epithelial mesenchymal transformation denotes the conversion of epithelium cells into mesenchyme cells under normal or special physiologic conditions [18]. Studies have shown that epithelial-mesenchymal transformation is vital for the modulation of malignancies, and Twist, Snsnail, N-cadherin, Vimentin, and E-cadherin are pivotal transcriptional factors that regulate the process of epithelial-mesenchymal transformation and are vital for embryo development and tissue genesis [19] Zhang Y, Zhang Y, Zhang Y, et al. Epithelial-mesenchymal transformation is an early marker of tumor invasion and metastases [20]. Herein, our team finally verified the roles of miR-339-5p in E-M transformation in human glioma U87 cells. The outcomes revealed that overly expressed miR-339-5p repressed the protein expression levels of Twist, Snsnail, N-cadherin, and Vimentin, facilitated the expression level of E-cadherin, suppressed the expression level of miR-339-5p, elevated the protein expression levels of Twist, Snail-2, N-cadherin, and Vimentin, but reduced the protein expression level of E-cadherin. Related research has unveiled that the transfection process of miR-339-5P mimics reduced the proliferative, migratory, invasive abilities, and other abilities of prostate carcinoma cells, increased apoptosis rate, increased E-cadherin in epithelial mesenchymal transformation, and decreased snell-2 and N-cadherin expression [21]. Other research has unveiled that miR-339-5P suppresses metastases of non-small-cell carcinoma via modulating E-M transformation [22], like the results of this study.

In summary, 49 gliomas were preliminarily screened out in this study. The expression of miRNAs is significantly different between glioma and healthy samples. The low expression level of miR-339-5p in glioma can modulate the proliferative, apoptotic, invasive, and migratory of glioma U87 cells and might exert an effect on tumor suppression during the occurrence and development of glioma.

## Figures and Tables

**Figure 1:** Heat map of miRNA microarray results in glioma brain tissue and normal tissue. Note: green denotes low expression level of miRNA, and red denotes high expression level of miRNA.

**Figure 2:** Expression of miRNAs in healthy and glioma samples.

**Figure 3:** Comparison of proliferation capability of human glioma U87 cells in each group. Note: in contrast to miR-NC group, ^a^*P* < 0.05 and ^b^*P* < 0.05 vs. mir-339-5p mimic group.

**Figure 4:** Apoptosis of human glioma U87 cells in all groups. Note: in contrast to miR-NC group, ^a^*P* < 0.05 and ^b^*P* < 0.05 vs. miR-339-5p mimic group.

**Figure 5:** Comparison of invasion capability of human glioma U87 cells in each group. Note: in contrast to miR-NC group, ^a^*P* < 0.05 and ^b^*P* < 0.05 vs. miR-339-5p mimic group.

**Figure 6:** Comparison of migration ability of human glioma U87 cells in each group. Note: in contrast to miR-NC group, ^a^*P* < 0.05 and ^b^*P* < 0.05 vs. miR-339-5p mimic group.

**Figure 7:** Expression of E-M transformation-related proteins in human glioma U87 cells of each group.

**Table 1:** Differential expression of miRNAs in glioma brain tissue.

Upregulated miRNA (*n* = 16)	Downregulated miRNA (*n* = 33)	
hsa-miR-10b-5p	hsa-miR-339-5p	hsa-miR-143-5p
hsa-miR-143-5p	hsa-miR-185	hsa-miR-23b-3p
hsa-miR-218-5p	hsa-miR-539	hsa-miR-455-5p
hsa-miR-133a	hsa-miR-454-3p	hsa-miR-140-3p
hsa-miR-93a	hsa-miR-323	hsa-miR-127
hsa-miR-16	hsa-miR-452-3p	hsa-miR-130a-3p
hsa-miR-30a	hsa-miR-95	hsa-miR-451
hsa-miR-517-5p	hsa-miR-126-3p	hsa-miR-96-5p
hsa-miR-339-5p	hsa-miR-382-5p	hsa-miR-498
hsa-miR-602	hsa-miR-126-3p	hsa-miR-505-5p
hsa-miR-409-3p	hsa-miR-495	hsa-miR-17-5p
hsa-miR-708-3p	hsa-miR-181a-5p	hsa-miR-221-5p
hsa-miR-517-5p	hsa-miR-21-5p	hsa-miR-181b
hsa-miR-365a-5p	hsa-miR-23b-3p	hsa-miR-181b
hsa-miR-6512-5p	hsa-miR-143-3p	hsa-miR-181c
hsa-miR-31	hsa-miR-4646-3p	hsa-miR-143-3p
	hsa-miR-145-5p	

## Data Availability

The data used to support the findings of this study are available from the corresponding author upon request.
